# A Multicultural Demographic Study to Analyze Antibiotic Prescription Practices and the Need for Continuing Education in Dentistry

**DOI:** 10.1155/2021/5599724

**Published:** 2021-07-16

**Authors:** Mohmed Isaqali Karobari, Shahnawaz Khijmatgar, Rahul Bhandary, U. S. Krishna Nayak, Massimo Del Fabbro, Rithvitou Horn, Anand Marya

**Affiliations:** ^1^Conservative Dentistry Unit, School of Dental Sciences, Universiti Sains Malaysia, Health Campus, 16150 Kubang Kerian, Kota Bharu, Kelantan, Malaysia; ^2^Department of Conservative Dentistry & Endodontics, Saveetha Dental College & Hospitals, Saveetha Institute of Medical and Technical Sciences University, Chennai 600077, Tamil Nadu, India; ^3^Department of Biomedical, Surgical and Dental Sciences, University of Milan, Italy; ^4^Nitte (Deemed to Be University), AB Shetty Memorial Institute of Dental Sciences, Department of Oral Biology and Genomic Studies, Mangalore, India; ^5^Nitte (Deemed to Be University), AB Shetty Memorial Institute of Dental Sciences, Department of Periodontics, Mangalore, India; ^6^Nitte (Deemed to Be University), AB Shetty Memorial Institute of Dental Sciences, Department of Orthodontics, Mangalore, India; ^7^IRCCS Galeazzi Orthopedic Institute, Via Riccardo Galeazzi, 4, 20161 Milano, Italy; ^8^Faculty of Dentistry, University of Puthisastra, Phnom Penh, Cambodia; ^9^Department of Orthodontics, Faculty of Dentistry, University of Puthisastra, Phnom Penh, Cambodia; ^10^Department of Orthodontics, Saveetha Dental College, Saveetha Institute of Medical and Technical Sciences, Saveetha University, Chennai, India

## Abstract

**Objectives:**

The objective of the study was to understand and analyze the prescription patterns of dentists across various demographic locations for managing oral infections and pain with antibiotics and explore the evidence-based practices by clinicians as well as the need for further education. *Materials and methods*. This cross-sectional study was carried out using an online questionnaire framed to explore the knowledge, attitude, and practices among dentists with varying levels of experience and qualifications, regarding antimicrobial prescription. The questions were validated from previous published studies that explored the knowledge, attitude, and practice (KAP) with respect to antimicrobial prescription. In total, *N* = 300 of dentists from four different countries responded to the online questionnaire out of which 53% were specialists while 47% were general dentists. After data collection, descriptive analysis was carried out along with a one-sided hypothesis test to depict the power of the sample.

**Results:**

It was seen from the results of the study that the first-choice antibiotics for 67.8% of dentists were found to be the *β*-lactam group while sulfonamides and tetracyclines at 20% were the second most prescribed group. Another important finding was that 45.6% of dentists ignored hypersensitivity testing before prescription of antibiotics even though 83.3% of the total dentists interviewed were aware of the increase in antibiotic resistance.

**Conclusion:**

In conclusion, the dentists are partially aware of the guidelines but need further training and education on antimicrobial prescription that enables evidence-based decision-making for better practices and outcomes.

## 1. Introduction

Antibiotics have been used extensively for both treatment as well as intervention for managing 1.7 million severe sepsis infections occurring each year [1]. Since antimicrobial prescription is influenced by various factors like systemic disease condition and prophylaxis to tackle the antimicrobial resistance (AMR), majority of the research in past few decades were focused on AMR, isolating new infection causing pathogens and identification of diseases [2]. In routine dental practice, bacterial infections are seen commonly and treated frequently with antibiotics. It was seen in previously conducted studies that odontogenic infections account for almost 10 percent of antibiotic usage in a year [3]. Over the past few years because of the enhanced use of antibiotics, there has been a corresponding increase in AMR. While antibiotics are essential for treatment of many infections, the inadvertent use of antibiotics by oral healthcare professionals has become a major cause of concern [4]. Approximately 700,000 people die because of antibiotic resistance in a calendar year, and this figure is only bound to increase with time [5]. There have been studies conducted on the use of antibiotics in the oral healthcare sector but the prescription practices across various regions have not been studied in detail. If dental practitioners are investigated for their prescription practices, then it would help understand and answer some of the questions regarding the rise of cases with AMR [6, 7]. In dentistry, prescription of antibiotics is most often due to tooth pain i.e., reversible and irreversible pulpitis or due to swelling. Antibiotics are prescribed by dentists for a period of 5-7 days, and these are accompanied by anti-inflammatory drugs for management of pain associated with the infection [8]. In a previous study, it was concluded that although penicillins are most commonly used for the management of odontogenic infections, the increase in penicillin-resistant strains of bacteria has led to use of other antibiotics such as clindamycin [9]. The most common uses of antibiotics in dentistry are in relation to odontogenic and nonodontogenic infections, prophylactic management in patients at risk of or with preexisting systemic disorders, management of local infections, and postsurgery or extractions.

In the United States, it has been seen that dentists with varying levels of specialization prescribe one-third of the entire quantity of antibiotics used in the country [10]. Additionally, studies conducted in the last 3 years have shown that around 30% of the antibiotics prescribed for dental problems were not indicated or required [11, 12]. Even though many countries have groups and associations that have listed recommendations for the judicious use of antibiotics for odontogenic and nonodontogenic infections, there have been guidelines established for these [13, 14]. The American Dental Association has recently published a set of guidelines and regulations for the management of pulpal and periapical oral problems using antibiotics [15].

While there are proven benefits of treatment of infections with antibiotics, there are associated reactions and side effects as well. It was seen that the development of bacterial resistance is a matter of concern, and the principal reason was increase in the occurrence of *β*-lactamase producing bacteria in odontogenic infection [16]. This is why there must be sound rationale behind the use of antibiotics which can help decrease the side effects as well as lower the increasing antimicrobial resistance.

In recent years, there have been studies conducted in developing countries such as India, Saudi Arabia, and Malaysia where it has been shown that the antibiotic prescribing practices were exceedingly flawed [17–20]. These studies also concluded with the obvious need for educational programs and initiatives that could help rationalize the use of antibiotics by dental practitioners. However, there is an urgent need to understand how clinicians make decisions and also to explore how the scale of evidence is translated into clinical practice. This is one of the reasons why dentists from these countries were included in a multicultural study to understand in detail the cause of concern.

Therefore, the objective of this survey was to identify the gaps in knowledge, attitude, and practices among dental practitioners in antimicrobial prescription and explore the evidence based practices among dentists.

## 2. Methodology

### 2.1. Site and Settings

The questionnaire was developed at Nitte (Deemed to be University) AB Shetty Memorial Institute of Dental Sciences, Department of Oral Biology and Genomic Studies, Mangalore, India. The questions were selected from previous evidence-based publications on knowledge, skills, and practice-associated outcomes [20–26]. The questionnaire was validated by distributing it among 20 dentists (Content experts) in the institute initially, and following validation, it was distributed online among dentists from four countries by (Mohmed Isaqali Karobari) MIK, (Shahnawaz Khijmatgar) SK, and (Anand Marya) AM via emails containing links to the Google survey [27, 28]. The university ethics committee reviewed the study protocol and confirmed that ethical approval was not required for this study.

### 2.2. Questionnaire

An online questionnaire was developed using Google survey to collect demographic data and study antibiotic prescription in practice using criteria such as qualifications, experience, location of practice, reasons for prescription, and commonly used antibiotics. No identifying data was collected at any point in the study. Also, a discretion statement was included in the questionnaire for the participants. Detailed information was collected on the purpose of antibiotic prescription, knowledge of protocols, and awareness of culture sensitivity and drugs to avoid in cases with liver or renal problems, superinfections and their management, antibiotics of choice, and duration as well as frequency.

### 2.3. Subjects

The dental practitioners were based in India, Malaysia, Saudi Arabia, and Cambodia. Licensed dental practitioners with work experience of more than a year were selected for this study. The researchers provided the online links to the questionnaire making use of Google survey, and nonqualified dental professionals and dentistry students were excluded from the study. The criteria for exclusion from the data collection were nonlicensed dental practitioners, licensed dental practitioners with less than one year of experience, dentistry students, dental hygienists, and dental technicians.

### 2.4. Bias

The questionnaires were designed based on previous evidence-based research that enabled participants in the study to answer questions related to antimicrobial prescription practices (psychometric tested questionnaires). Other factors that were considered: planning the content, questionnaire layout and order, piloting (piloting done at the study setting location), response rate, and considering the content validity of the questions.

### 2.5. Statistics

A descriptive statistical analysis, sample size calculation, and significance were identified using STATA/IC 16.1 statistical software. For analysis, descriptive statistics of the sample size were prepared, and the numerical data was tested for association between the sample size and the population size (Figure 1). The sample size analysis was carried out in this study to ascertain that a study sample of 100 dentists would be optimal to achieve the research objectives of the study. As can be seen from the results of the sample size analysis, a study sample of approximately 300 dentists is enough to represent a dental population size of 6000 dentists, thus making the outcome of the study successful. The one-sided hypothesis test also asserted that the target sample for the sample taken for the study was enough to get an optimal outcome (Figure 2).

## 3. Results

The online questionnaire contained demographic information such as qualifications, years of experience, and types of practice. Data was collected from participating dentists regarding their patterns of antibiotic prescription across various clinical scenarios and problems. The dentists were also asked to divulge their most prescribed antibiotics in patients reporting to their clinics with different odontogenic and nonodontogenic problems. The response rate was 90.9%.

Out of a total of *N* = 350 of dental practitioners that were sent in the online questionnaire, *N* = 318 of dentists responded by completing and answering all questions that were asked. Of the *N* = 318 of dentists that answered, 18 responses were excluded for reasons such as not completing the entire form or location not from the area under focus. From the 300 dentists that were included as part of the sample, 53.3% were general dentists, and 46.7% were dentists with specialist qualifications (Figure 3(a)). Among the total respondents, 22.2% of dentists had 20 years of experience or more, and 60% of dentists had less than 5 years of experience (Figures 3(b) and 3(c)). When further information was asked regarding qualifications, 42.2% of respondents revealed that they had a general dentist qualification with no additional certifications, 34.4% had graduated from an accredited master's program, and 13.3% held an overseas qualification in addition to their basic qualification.

Regarding antibiotic usage, 58.9% of dentists responded that they would prescribe antibiotics for odontogenic infections, periodontal infections, dentoalveolar trauma, and prophylactic coverage. 27.8% of dentists responded that in addition to the previously mentioned criteria, they would prescribe antibiotics for management of other problems such as nonodontogenic infections, following routine extractions, etc. (Figure 4(a)). For extractions, 63.3% of dentists would avoid prescribing antibiotics after every extraction while 24.4% of dentists would prescribe antibiotics after every tooth extraction and 12.2% of dentists responded by answering that they would use antibiotics selectively (Figure 4(b)).

While 20% of dentists out of the total would prescribe antibiotics prior to oral surgical procedures in nonmedically compromised patients, 26.7% of dentists would do so depending on the procedure to be carried out while 52.2% of respondents avoided antibiotic prescriptions in noncompromised cases (Figure 4(c)). A vast majority of dentists, i.e., 57.8%, did not routinely prescribe broad-spectrum antibiotics in contrast to 31.1% of dentists that did so while 11.1% of dentists only used them depending on the case (Figure 4(d)). The first-choice antibiotics for 67.8% of dentists were found to be the *β*-lactam group while sulfonamides and tetracyclines at 20% were the second most prescribed group. Aminoglycosides and macrolides at 16.7% were the third most popularly prescribed antibiotics with nitrofurans, lincosamides, and glycopeptides not being used at all.

Prophylactically 45.6% of dentists used a combination of amoxycillin with clavulanate while plain amoxycillin was the antibiotic of choice for 43.3% of respondents with cephalosporins the third in the order (Figure 5(a)). It was seen that 85.6% of dentists interviewed followed standard protocols for duration and dosage for antibiotics while 10% would prescribe these medicines on a case-to-case basis (Figure 5(b)).

The need for prescribing antibiotics was also questioned with 87.8% of dentists using antibiotics for spreading infections, 55% for lymphadenitis, and another 50% for localized swelling. Routine dental procedures such as scaling did not warrant the use of antibiotics; so, 83.3% of dentists would avoid prescribing antibiotics, similarly for subgingival restorations at 68.9% and impressions at 90%. Patients receiving endodontic treatment were not given antibiotics by 34.4% of dentists while only 20% of dentists avoided giving antibiotics for routine extractions. An interesting finding was that 26.7% of dentists were found to prescribe antibiotics for pulpitis while another 42.2% responded that they would selectively. Only 30% of dentists said that they would avoid giving antibiotics in case of pulpal involvement (Figure 6(a)). 75.6% of dentists were aware of the list of drugs to avoid in case of liver or renal problems while 15.6% of dentists were not sure (Figure 6(b)). The importance of culture sensitivity testing was shown to be neglected by 76.7% of dentists who prescribed antibiotics without it while 17.8% of respondents said they could get it done (Figure 6(c)). Another important finding was that 45.6% of dentists did not test the patient for hypersensitivity before prescription of antibiotics and only 14.4% of dentists replied in the affirmative even though 83.3% of the total dentists interviewed were well aware of the increase in antibiotic resistance (Figures 1(a) and 6(d). 67.8% of the study sample never encountered superinfection in a patient who was administered antibiotics which is also the reason that 28.9% were not even aware of the management protocols for the same (Figure 1(b)).

Patient negligence in terms of self-medications was also noticed by 76.7% of dentists while 82.2% of oral health professionals replied in the negative when they were asked if they prescribed medicines at the insistence of the patients (Figure 1(b)). The final question was regarding the influence of nonclinical factors, and 72.2% of dentists responded that they would prescribe antibiotics for patients who wished to delay elective treatment procedures while a surprisingly high number, i.e., 32.2% of dentists provided patients with a prescription for antibiotics even when they were uncertain of the diagnosis (Figure 1(b)).

## 4. Discussion

Antibiotic therapy has been a vital part of dentistry since the past few decades. The ever-increasing problem is that while dentists routinely engage in skill-based learning, a similar effort is not devoted to understanding and adapting the latest clinical guidelines on antibiotic prophylaxis to their practice. This attitude may be due to the lack of awareness about importance of evidence-based guidelines, time constraints, and resources required and lack of training. As can be seen from the abovementioned results, dentists routinely engage in empirical antibiotic prescription and at times neglecting the serious side effects that may result from the inadvertent use of these medicines (Figures 1(b) and 6(a)). Dentists responded they would prescribe antibiotics in cases of pulpitis. An attempt must be consciously made to reduce misuse of antibiotics and prevent the further growth of antimicrobial resistance. While drug resistance maybe a natural phenomenon, what dentists must focus is on acquired antimicrobial resistance that can develop because of misuse of antibiotics [29]. Dentists have been prescribing medicines for pain in cases such as irreversible pulpitis, but this is neither recommended nor effective as has been shown in previous studies [30].

One of the main problems faced regarding antibiotic usage is the lack of clear guidelines for their prescription [31], which was the case in the past. But recently, new guidelines have been developed. Dental pulp infections are routinely caused by microorganisms; however, not all cases indicated for endodontic management require antibiotics if the pulp chamber is completely debrided followed by obturation and sealing of the root apex [32]. The only way of determining the effectiveness of a prescribed antibiotic is an improvement in the symptoms of the patient [33]. According to the British Society for Antimicrobial Therapy, inappropriate and inadvertent use of antibiotics brings about an increase in antibiotic-resistant strains compared to their susceptible population thereby leading to resistance. This rise of resistant strains invariably contributes to a greater rise in the mortality rates resulting from infections [34]. It was seen in this study that almost 26 percent of the dentists investigated prescribed antibiotics for management of pulpitis which was much higher compared to other studies [35]. More than half of the dentists that answered the questionnaire preferred the use of beta-lactam antibiotics which falls in accordance with results from other studies [36].

Some distressing issues that were noticed were that some dentists, i.e., 18.9% would prescribe antibiotics for nonclinical factors such as postponing procedures and even on the patient's insistence which was in accordance with studies conducted [37]. 24.4% of dentists were found to routinely prescribe moderate doses of antibiotics following extractions only to avoid posttreatment complications [37]. The study was carried out with dentists having varying levels of experience to understand whether there was a definite correlation between the experience and prescribing practices but there was none. A concerning finding of this study is the lack of educational programs focusing on antibiotic prescription practices leading to the current situation. Some of the limitations of our study were not having additional sections on managing consultations, postextraction infections, or questions on existing location-based guidelines. This was solely because our focus was on evaluating current prescription practices and analyzes associated problems.

Antibiotics must be studied in detail in terms of microbiology, epidemiology, infection control, indications, and contraindications as well as pharmacology of each specific drug. To ensure antibiotics are prescribed properly, the aforementioned factors must be understood so that antimicrobial resistance can be brought under control. There are immunocompromised patients as well as patients with systemic disorders that must be given antibiotic prophylaxis in consultation with their treating physician. It is also seen that there are a lot of dental procedures in which antibiotics are not required which reaffirm the fact that these must be considered adjunctive to the treatment modality. A recent study on galectin role (increasingly secreted by macrophages) in managing oral health was reported [38]. The findings of the study demonstrated antimicrobial activity towards pathogenic organisms like Candida albicans among other pathogens that present in the oral biofilm, thus revealing an interesting therapeutic role of galectin and other biomarkers [39], but to translate these findings into clinical practice would require clinicians having a detailed understanding the important role of galectin. Faculties at higher education institutions should train graduates and postgraduates taking innovation and new findings into account when carrying out clinical practice.

Many of the findings of the study confirm findings from previous studies conducted across India, Malaysia, and Saudi Arabia that reported an excess use of antibiotics in situations where they may not be required [17, 18]. Our study found that broad-spectrum antibiotics especially were being overprescribed in situations where they were not required such as irreversible pulpitis. This could be attributed to a lack of knowledge or a relaxed attitude towards gaining education regarding the latest guidelines and practices.

Dentists that prescribe antibiotics for dental or oral infections must evaluate patients on a routine basis and as soon as an improvement in the patient's symptoms is seen in the antibiotic therapy should be terminated. As can be seen from the results of this study, there is widespread inconsistency regarding the prescription, duration, and need for prescribing antibiotics. Therefore, efforts must be made to improve the attitude and knowledge of all dental practitioners to ensure that uniform prescription patterns are established leading to a selective use of antibiotics only in conditions where they are required. It has been seen that the bacterial strains found in the oral cavity are becoming increasingly resistant as well as newer more resistant strains are being detected.

### 4.1. Limitations

There is lack of larger and more regional sample sizes to evaluate the knowledge, attitude, and practice of dentists regarding the use of antibiotics.

There is lack of input from the governing authorities regarding their current educational programs on antibiotic prescription practices.

There is lack of information on how many programs dentists are attending to learn about antibiotics and where to prescribe.

## 5. Conclusion

In conclusion, dental practitioners made prescription decisions to delay the elective procedures followed by uncertain diagnosis. Majority of dentists faced self-medication by patients given by pharmacists upon patient requests. There is still confusion among dentists whether to give antibiotics in cases of pain and pulpitis; although, there are guidelines and evidence published in this regard. There is clear lack of transforming evidence-based information into clinical practice. One of the possible reasons may be is that there is lack of communication or gaps between basic research, clinical research, clinicians, policy makers and reformers, societies, councils and lastly, pharma industry. In addition, there is a need of training in antimicrobial prescription for dentists when they qualified and recommend respective dental councils to implement mandatory continuing professional development. Also, increase in awareness among patients regarding antimicrobials and antimicrobial resistance is a need.

### 5.1. Recommendations

Based on the findings of this study, we would like to offer the following recommendations:

1. More efforts need to be directed at educating general dental practitioners, new specialists, and faculties about the evidence-based guidelines in antibiotic prescription
2. Organization of educational and training programs should train newly graduating dentists and postgraduates to educate them about the latest prescription guidelines and to create more awareness about the rise in antimicrobial resistance
3. Continuous evaluation of prescribing practices to ensure uniform delivery of antibiotics and taking pharmacist on board. Also, making conscious efforts to slow down the rise of antibiotic-related problems that arise during clinical practice

## Figures and Tables

**Figure 1:** (a) Have you ever encountered superinfection in a patient following antibiotic prescription? (b) Are you aware of the management protocol for the treatment of superinfections?

**Figure 2:** Calculation of the sample size and its representation.

**Figure 3:** (a) Types of dental practice. (b) represents the work experience of the participating dentists in years. (c) Graphical representation of the percentage of the year of graduation of the participating dentists.

**Figure 4:** (a) Which conditions do you most often prescribe antibiotics for? (b) Do you prescribe antibiotics following every extraction? (c) Do you prescribe antibiotics prophylactically prior to oral surgical procedures in nonmedically compromised patients? (d) Do you routinely prescribe antibiotics?

**Figure 5:** (a) Which drug do you prescribe most for the purpose of prophylaxis? (b) Do you follow standard protocols for dosage and duration when prescribing antibiotics?

**Figure 6:** (a) Would you prescribe antibiotics for pulpitis?. (b) Do you test for culture sensitivity prior to antibiotic prescription? (c) Have you encountered self-medication of antibiotics amongst your patients? (d) Are you aware of the rise in antibiotic resistance?

## Data Availability

Any data related to the study can be provided on reasonable request.
